The article "Quality Evaluation of Ideological and Political Education in Universities Based on BP Neural Network" was retracted in 2023. Reasons: unreliable results or conclusions; concerns about the data; concerns about the peer review; concerns about the citations.

# Quality Evaluation of Ideological and Political Education in Universities Based on BP Neural Network

**DOI:** 10.1155/2022/8336895

**Published:** 2022-07-18

**Authors:** Yunxia Ding, Wei Zeng, Zhen Ning

**Affiliations:** Jiangxi University of Technology, Nanchang 330098, China

## Abstract

At present, there are some problems in the research of curriculum ideological and political quality evaluation, such as insufficient theme attention, insufficient theoretical research, incomplete data collection, and so on. This study aims to use the BP neural network in the ideological and political quality evaluation system so that the system can more comprehensively and accurately reflect the actual situation of students and point out the direction for the development of students' ideological and political education. The construction of this system can provide a very considerable and accurate way for the quality evaluation of ideological and political education of college students and especially solves the problems of human subjective, factor errors, and the setting of evaluation index weights in the evaluation system.

## 1. Introduction

Since the reform and opening up, the reform of ideological and political theory classroom teaching in universities nationwide has been continuously going on, although great achievements have been made. However, the reform of classroom teaching of ideological and political theory course has been concentrated on teaching content and curriculum, while the reform of classroom teaching index system evaluation of ideological and political theory course seems to be rather lagging behind [1–3]. The so-called teaching quality evaluation is to assess the standard, efficiency, and quality of teaching activities according to the teaching objectives, and to estimate and judge the value of teaching. The talent training effect is the primary standard for the evaluation of curriculum ideological and political construction. It is necessary to establish and improve the multidimensional evaluation system and supervision and inspection mechanism of curriculum ideological and political construction effect, and implement it in all kinds of evaluation work and deepen the reform of education and teaching in colleges and universities.

Although many teachers engaged in teaching ideological and political theory courses also attach great importance to the research and summary of teaching experience and methods, the research results of the classroom teaching evaluation index system with weight are rare. Based on the above analysis, how to improve the teaching level and quality of ideological and political theory courses in universities, the study of classroom teaching evaluation index and its system is fundamental to improve the level and quality. Therefore, the construction of a curriculum ideological and political quality evaluation system is of great significance. It is the guarantee measure to promote the full implementation of curriculum ideological and political education, the measurement standard to test the quality of curriculum ideological and political teaching, and the feedback mechanism to improve the effectiveness of curriculum ideological and political education.

This study is the first attempt to use the BP neural network modeling to evaluate the effectiveness of online ideological and political education in universities. The research results show that the BP neural network can effectively improve the precision of college ideological and political classroom teaching quality evaluation and provide a new method and way for college ideological and political classroom teaching quality evaluation.

## 2. Features of BP Neural Network Model

The artificial neural network model does not require any a priori formula and has the advantages of self-learning, self-organization, self-adaptation, good fault tolerance, and strong nonlinear mapping ability, which is especially suitable for the processing of pattern recognition, data mining, and classification problems with complex variables and relationships.

The BP neural network is the most widely used artificial neural network algorithm, and the characteristics of the BP neural network model are as follows: each layer neuron is only connected with the neighboring layer neuron; there is no connection between neurons in each layer; and there is no feedback connection between neurons in each layer. The learning process is characterized by two parts: forward propagation of data and backward propagation of error, and the most suitable network model for the sample is built by continuously reducing the error. The BP neural network has infinite approximation of nonlinear mapping capability, powerful parallel processing capability, self-learning, self-organization and self-adaptability, data inclusion capability, and effective complex variable processing capability, which is especially suitable for multivariate function simulation, pattern recognition, judgment, classification, data processing, and other problems.

The BP neural network model is currently widely used in various disciplines. Wang [4] proposed a general public budget revenue forecasting analysis model based on gray forecasting and BP neural network and applied it in the case of Wuxi city. Ma [5] evaluated the effectiveness evaluation of online ideological and political education in colleges and universities based on the BP neural network. Wu et al. [6] studied the error compensation for airborne laser ranging based on the BP neural network. Lee et al. [7] integrated a cloud-based BP system with CPOE to improve self-management of the hypertensive patients and carried out a randomized controlled trial. These existing studies provide a reference for the work of this study.

## 3. The Problems of the Traditional Evaluation System of Ideological and Political Education in Universities

### 3.1. Single Evaluation Subject

Nowadays, the evaluation system of teachers' teaching quality is commonly carried out in all universities in China, such as students' evaluation of teachers, peer evaluation, administrative leaders' evaluation, experts' evaluation, and teachers' self-evaluation. The subjects of evaluation are students, peer teachers, administrators, and teachers' self-evaluation, which are usually evaluated by some combination of these four evaluation subjects, each of which has its own advantages and disadvantages. No matter which evaluation method is used, it is a one-sided evaluation with limitations, while teachers' teaching activity is a comprehensive activity with complexity and creativity.

### 3.2. Incomplete Evaluation Indicators

The teaching quality evaluation index is what evaluation index is the angle or dimension of measuring things. At present, most higher educational institutions in China have established a teaching quality evaluation index system, and the evaluation content versions of each university are similar, including teaching methods, teaching attitudes, teaching effects, and other aspects. The content of the evaluation is relatively simple, as if classroom theoretical teaching is all the evaluation of teaching quality. Some important contents, such as practical training teaching, engineering practice ability, students' comprehensive quality, and whether the specification and quality of cultivated talents meet the needs of the society, are excluded from the evaluation scope, forming a narrow object of teaching evaluation and a flat object coverage, which cannot comprehensively reflect the teaching quality.

### 3.3. Distortion of Evaluation Results

In recent years, the participation of college students as the main body in teachers' teaching evaluation has become a common way of teaching evaluation in China's universities. As the direct objects of classroom teaching, students have the most detailed understanding and deepest feelings about teachers' teaching attitude, teaching level, teaching effect, and teachers' moral standards, so they have the most right to evaluate. However, it is a long-standing controversial issue whether students, as the main subjects of teaching quality monitoring and evaluation, are objective and credible in their evaluation results. Those who resist and oppose are mainly from teachers, and there are many good teachers. There are two main reasons for this: one is that good teachers with strong dedication, strict requirements for students, and never “accommodating” students in examination results are not “well-rewarded,” and the other is that they are worried that it will mislead teachers to lower their requirements for students and cater to and accommodate students, which will have a negative impact on teaching quality. The practice of teaching quality monitoring and evaluation proves that these two tendencies do exist, and to a certain extent, they also distort the results of teaching quality monitoring and evaluation.

## 4. Construction of the Evaluation System of Ideological and Political Education Quality in Universities Based on BP Neural Network

### 4.1. Teachers' Teaching Quality Evaluation Index System

The evaluation index system refers to an organic whole with an internal structure composed of multiple indexes representing the characteristics of all aspects of the evaluation object and their interrelations. There must be a certain logical relationship between each index. They should not only reflect the main characteristics and states of each subsystem from different aspects, but also reflect the internal relationship between each subsystem. Each subsystem is composed of a group of indicators, which are independent and connected with each other to form an organic unity. The construction of the index system is hierarchical, from top to bottom, from macro to micro, forming an inseparable evaluation system.

Teaching quality evaluation must first determine a scientific teaching quality evaluation index system. In this study, based on the in-depth interviews with some teachers and students of a university and the summary of teaching quality evaluation research theories and practices in higher educational institutions at home and abroad, a comprehensive evaluation index system of teachers' teaching quality in various aspects such as teachers' teaching prerequisite factors, teaching process, and teaching effect is constructed (Table 1).

### 4.2. Teaching Quality Evaluation Model and Application

#### 4.2.1. Evaluation Model Construction

From the evaluation index system of teaching quality of university teachers, it can be seen that the factors affecting their teaching quality mainly include four categories of teaching prerequisites, such as teachers' commitment and responsibility to teaching, teachers' education and teaching ability, teachers' subject knowledge quality, and teachers' scientific research achievements and scientific research ability. The factors involved in the teaching process are six categories: the scientificity of the teaching contents and the amount of effective information contained in them, the reasonableness of the teaching methods, the cultivation of students' interest in learning, the appropriateness of the teachers' professional personality and teaching characteristics, the adaptability of the teaching contents to the students' needs, and the teachers' compliance with the school's teaching regulations and discipline. The improvement of students 'political thought and moral quality, the acquisition of students' basic professional knowledge and general knowledge, and the improvement of students' practice and self-development ability are represented as *I*_11_, *I*_12_, *I*_13_, *I*_14_, *I*_21_, *I*_22_, *I*_23_, *I*_24_, *I*_25_, *I*_26_, *I*_31_, *I*_32_, *I*_33_. If the teaching quality evaluation process of university teachers is modeled as a BP neural network system, the system is studied by taking teaching quality as the output of the system and all the influencing factors affecting teaching quality as the input of the system (multiple inputs).

The BP network is a hierarchical feedforward neural network consisting of an input layer, intermediate layer, and output layer. The intermediate layer can be extended into multiple layers; the neurons are connected between adjacent layers and within the same layer according to a certain structure; and the learning training is conducted in the way the teacher shows and teaches to determine the threshold value of each neuron and the weight value between each neuron, so that the neural network has a certain “function” or “intelligence.” However, the BP neural network itself has some defects and shortcomings, mainly including slow convergence speed, easy to input local minimal, difficult to determine the appropriate number of hidden layers and hidden nodes, and poor prediction effect on data with large numerical quantity relationship [6–9]. To address the shortcomings of “slow convergence speed” and “poor prediction for data with large numerical relationships,” the standard BP algorithm (i.e., absolute error backpropagation algorithm) is improved by applying the relative error of the data as the error signal. This study applies the relative error of data as the error signal to improve the standard BP algorithm (i.e., absolute error backpropagation algorithm) in order to improve the accuracy of the BP neural network. For establishing the neural network model with the function of “university teaching quality evaluation,” this study adopts the “three-layer” BP network, the number of neurons in the first input layer (13 evaluation indexes affecting its teaching quality) is 13, the number of neurons in the second intermediate layer is 28, and the number of structural neurons in the third layer is 28. The number of neurons of the third output layer (teaching quality) is 1. The BP network [10–14] is trained by using the teaching quality evaluation data to find out the correlation between the teaching quality and the evaluation indexes of university teachers. Then, they further rely on the trained BP network to calculate the teaching quality of teachers under different influencing factors (each evaluation index).

The specific learning training algorithm is implemented as follows:

(1) *N* sets of training samples from the teaching quality evaluation data are selected as the BP network input and output samples for training, and the remaining data are used as the test samples. For the *k*th sample, we set the BP network input pattern vector *U*^*k*^=(*u*_1_^*k*^, *u*_2_^*k*^,…, *u*_*s*_^*k*^) (*s* is the number of neurons in the network input layer 13) corresponding to the desired output vector *X*^*k*^=(*x*_1_^*k*^, *x*_2_^*k*^,…, *x*_*q*_^*k*^) (*q* is the number of neurons in the network output layer 1), the output layer unit input vector *M*^*k*^=(*m*_1_^*k*^, *m*_2_^*k*^,…, *m*_*q*_^*k*^), the output layer unit output vector *N*^*k*^=(*n*_1_^*k*^, *n*_2_^*k*^,…, *n*_*p*_^*k*^), the intermediate layer unit input vector *G*^*k*^=(*n*_1_^*k*^, *n*_2_^*k*^,…, *n*_*p*_^*k*^), the intermediate layer unit output vector *H*^*k*^=(*h*_1_^*k*^, *h*_2_^*k*^,…, *h*_*p*_^*k*^) (*p* is the number of intermediate layer neurons 28), input layer to intermediate layer connection weight is *H*^*k*^=(*h*_1_^*k*^, *h*_2_^*k*^,…, *h*_*p*_^*k*^), intermediate layer to output layer connection weight is *v*_*jt*_(*j*=1,2, ⋯, *p*; *t*=1,2, ⋯, *q*), intermediate layer unit threshold is *θ*_*j*_(*j*=1,2, ⋯, *p*), output layer unit threshold is *γ*_*t*_(*t*=1,2, ⋯, *q*), *η* is the learning rate, and network response function *f*(*x*) = 1/(1 + *e*^−*x*^).
(2) We assign the initial values of weights and thresholds *w*_*ij*_ (*n*), *v*_*jt*_ (*n*), *γ*_*t*_ (*n*), and *θ*_*j*_ (*n*) to random values in the interval [−1,1], and set *n* = 0 and *k* = 0.
(3) We set *k* = *k* + 1, assign the values of *I*_11_, *I*_12_, *I*_13_, *I*_14_, *I*_21_, *I*_22_, *I*_23_, *I*_24_, *I*_25_, *I*_26_, *I*_31_, *I*_32_, *I*_33_ of the *k*th set of sample data in the *N* sets of training samples to the elements *U*_1_^*k*^, *U*_2_^*k*^, *U*_3_^*k*^, *U*_4_^*k*^, *U*_5_^*k*^, *U*_6_^*k*^, *U*_7_^*k*^, *U*_8_^*k*^, *U*_9_^*k*^, *U*_10_^*k*^, *U*_10_^*k*^, *U*_12_^*k*^, *U*_13_^*k*^ in the input pattern vector *U*^*k*^, and assign the values of teacher teaching quality *I* to the elements *X*_1_^*k*^ in the output vector *X*^*k*^.
(4) According to equations (1) and (2), the actual outputs of the intermediate layer and the output layer are calculated as *h*_*j*_^*k*^ and *n*_*t*_^*k*^.
The output layer is as follows:
  (1) $$\begin{array}{c} \left\{\begin{array}{c} \text{input}:m_{t}^{k}=\sum_{j=1}^{p}v_{jt}h_{j}^{k}-\gamma_{t},\;\left(t=1,2,\ldots ,q;k=1,2,\ldots ,N\right),\\ \text{output}:n_{t}^{k}=f\left(m_{t}^{k}\right), \end{array}\right. \end{array}$$
  (2) $$\begin{array}{c} \left\{\begin{array}{c} \text{input}:g_{j}^{k}=\sum_{i=1}^{s}w_{ij}u_{i}^{k}-\theta_{j}\left(j=1,2,\ldots ,p;k=1,2,\ldots ,N\right),\\ \text{output}:h_{t}^{k}=f\left(g_{j}^{k}\right). \end{array}\right. \end{array}$$
(5) The steepest gradient descent method is used to learn multilayer error correction for the network. The standard BP algorithm usually uses absolute error as the error transfer signal in the process of calculating values, which often makes the error large. This is due to the fact that absolute error tends to invariably magnify the overall error value of the system without considering the relationship with the actual value, which results in less accurate and slower final prediction results. The use of relative error as the transmission signal of the BP neural network error can well avoid the impact of such shortcomings. That is, the absolute error in the standard BP algorithm (*x*_*t*_^*k*^ − *n*_*t*_^*k*^) is replaced by the relative error (*x*_*t*_^*k*^ − *n*_*t*_^*k*^), and the generalized error sum of each unit in the output and intermediate layers is calculated by using equations (3) and (4).
  (3) $$\begin{array}{c} d_{t}^{k}=\frac{\left(x_{t}^{k}-n_{t}^{k}\right)n_{t}^{k}\left(1-n_{t}^{k}\right)}{{\left(x_{t}^{k}\right)}^{2}},\;\left(t=1,2,\cdots ,N\right), \end{array}$$
  (4) $$\begin{array}{c} e_{j}^{k}=\left[\sum_{t=1}^{q}d_{t}^{k}\cdot v_{jt}\right]h_{j}^{k}\left(1-h_{j}^{k}\right),\;\left(j=1,2,\cdots ,p\right). \end{array}$$
(6) If *k* = *N*, then we go to equation (7); otherwise, we go to equation (4) to continue the execution.
(7) We correct the connection weights *v*_*jt*_ and thresholds *γ*_*t*_ with the generalized error of each unit in the output layer *d*_*t*_^*k*^ and the output of each unit in the intermediate layer *h*_*j*_^*k*^, as shown in equations (5) and (6); we correct the connection weights *h*_*j*_^*k*^ and thresholds *θ*_*j*_ with the generalized *error of each unit in the intermediate layere*_*j*_^*k*^*and the input of each unit in the input layer,U*^*k*^=(*u*_1_^*k*^, *u*_2_^*k*^, ⋯, *u*_*s*_^*k*^), as shown in equations (7) and (8); and we set *k* = 0.
  (5) $$\begin{array}{c} v_{jt}\left(n+1\right)=v_{jt}\left(n\right)+\eta \sum_{k=1}^{N}d_{t}^{k}h_{j}^{k}, \end{array}$$
  (6) $$\begin{array}{c} \gamma_{t}\left(n+1\right)=\gamma_{t}\left(n\right)+\eta \sum_{k=1}^{N}d_{t}^{k}, \end{array}$$
  (7) $$\begin{array}{c} \theta_{j}\left(n+1\right)=\theta_{j}\left(n\right)+\eta \sum_{k=1}^{N}e_{j}^{k}, \end{array}$$
  (8) $$\begin{array}{c} w_{ij}\left(n+1\right)=w_{ij}\left(n\right)+\eta \sum_{k=1}^{N}e_{j}^{k}u_{i}^{k}. \end{array}$$
(8) It is recalculated with the new weights and thresholds *h*_*j*_^*k*^*n*_*t*_^*k*^(*k*=1,2,…, *N*). According to the accuracy requirement, if for each*k*(*k*=1,2,3 … …*N*)and each*t*(*t*=1,2,3 … *q*)are satisfied: ‖*x*_*t*_^*k*^ − *n*_*t*_^*k*^‖〈*ε* (*ε*is apregiven precision and set *ε* = 10^−6^) then learning stops. Otherwise, we set *k* = 0, go to equation (4), and remodify the weights and thresholds until the error accuracy requirement is satisfied.
(9) Using the trained BP network [15–18], the values of *I*_11_, *I*_12_, *I*_13_, *I*_14_, *I*_21_, *I*_22_, *I*_23_, *I*_24_, *I*_25_, *I*_26_, *I*_31_, *I*_32_, *I*_33_ in the input test samples are assigned to the elements *U*_1_^*k*^, *U*_2_^*k*^, *U*_3_^*k*^, *U*_4_^*k*^, *U*_5_^*k*^, *U*_6_^*k*^, *U*_7_^*k*^, *U*_8_^*k*^, *U*_9_^*k*^, *U*_10_^*k*^, *U*_10_^*k*^, *U*_12_^*k*^, *U*_13_^*k*^ in the input pattern vector *U*^*k*^, and the values of the elements *n*_1_^*k*^ in the output vector, i.e., *N*^*k*^=(*n*_1_^*k*^, *n*_2_^*k*^,…, *n*_*q*_^*k*^), the value of teacher teaching quality *I*, are predicted by simulation.

#### 4.2.2. System Implementation and Application

In this study, a total of 30 students in different classes taught by teachers of two main courses in a university are used as the survey samples, and the surveyed students rate the teachers' performance on each subevaluation index and the overall situation of teachers' teaching quality, respectively. The scores for the overall situation of each index are 1 (poor), 2 (general), 3 (good), and 4 (excellent), corresponding to scores of 45, 60, 75, and 90, respectively.

Using the established evaluation model [17, 18] of university teachers' teaching quality, the first 25 sets of survey data were fitted to the designed evaluation model to solve the unknown parameters in the evaluation model, and the last 5 sets of survey data were used as the test sample data. The evaluation model with the determined parameters was used to calculate the data of the 25 groups of samples that participated in the modeling and the data of the 5 groups of samples that did not participate in the modeling. Combined with the evaluation model, the data were processed with the simulation software system for evaluating the teaching quality of college teachers developed by Microsoft Visual Studio based on the Windows 8 x64 platform, and the results shown in Table 2 are obtained. From the table, it can be seen that the results obtained by the teacher teaching evaluation model based on the optimized neural network are very good, and the relative error is less than 10%.

## 5. Suggestions for Optimizing the Effectiveness of Ideological and Political Teaching in Universities

### 5.1. Establish a High-Quality and High-Skilled Ideological and Political Science Teachers' Team

Cultivating teachers' comprehensive quality and establishing a high-quality and high-skilled civic and political science teachers' team are the main prerequisites for strengthening and improving the effectiveness of ideological and political teaching in universities under the new situation. Combined with the actual situation, ideological and political teachers first need to cultivate theoretical literacy, constantly enrich themselves on the basis of establishing the awareness of lifelong learning, learning advanced knowledge, paying attention to social hotspots, while keeping good contact with students, understanding students' confusion and needs, and helping them solve problems in time; second, they need to cultivate moral cultivation, use the method of linking theory to practice to teach students, and be a good role model for them. This method of using practical actions to educate students is more effective than purely theoretical teaching, and it is easy to gain students' recognition; finally, it is necessary to cultivate the educational ability, to play a variety of roles in teaching, such as organizer, guide, coordinator, and manager, to respect the main position of students, to create an equal and harmonious teaching environment, to strengthen practical teaching while focusing on theoretical teaching, and to further improve the relevance and effectiveness of teaching, and effectiveness.

### 5.2. Pay Attention to the Cultivation of Students' Sense of Identity in Ideology and Politics

Understanding students' needs and cultivating students' sense of identity in ideology and politics are important basis for strengthening and improving the effectiveness of ideological and political teaching in universities under the new situation. Students are the main body of classroom teaching, and today, with the continuous development of new curriculum reform, it has become the consensus of college education to play the main role of students and respect students' interests and demands. Compared with other courses, the ideological and political course has certain advantages in the propagation and learning of party policies. Teachers need to use this advantage to highlight the role and charm of the ideological and political course and inspire students to pay attention to the ideological and political learning. In addition, teaching ideology and politics is a practical subject, and when teaching in practice, it is necessary to combine students' interests and personality characteristics to design activities, and to cultivate students' healthy personalities while enjoying their body and mind. Therefore, civic teachers need to stimulate students' participation in practical teaching through multiple channels, give students more free time and space in the specific practice process, and guide them to use what they have learned to solve real-life problems, so that they can further realize the importance and necessity of ideological and political teaching and thus develop a sense of identity.

### 5.3. Reflect the Rationality and Scientificity of Teaching Objectives

The setting of teaching objectives is crucial for any lesson; ideological and political teaching in universities is no exception; and teaching objectives are the main basis for judging the degree of effectiveness of its teaching. Ideological and political teaching emphasizes the combination of theoretical and practical teaching, among which the setting and selection of practical teaching objectives have a direct impact on teaching content, teaching evaluation, and teaching form, and should be paid great attention. The general goal is the general goal of theoretical teaching, which is to improve students' understanding of the connotation and spirit of Marxism, their ability to apply Marxist concepts and methods, to establish correct learning concepts, to clarify their duties and obligations, and to take the initiative to learn and move forward in the direction of excellent socialist builders through participation in practical activities. It should be noted that the specific goal system should cover various aspects, such as knowledge, skills, and emotions.

### 5.4. Play the Role of Modern Media to Improve the Effect of Teaching Mode

In today's increasingly popular network, multimedia computers and other media gradually come into the life of college students, changing their learning style and thinking mode; multimedia computers and other media are new media in the background of the new situation; and there are certain differences with traditional media. The teachers of higher education need to compare the new media with the traditional media on the basis of understanding the characteristics of the new media, give the traditional media new connotation, and establish an interactive teaching method that meets the requirements of the new situation, so as to achieve the purpose of enriching the content of ideological and political teaching and improving the relevance and effectiveness of ideological and political teaching. Second, they need to respect students' main position, design teaching around students, and change students' passive acceptance into active learning; finally, they need to build an equal and harmonious teaching environment, and promote the realization of equality and dialogue among subjects.

### 5.5. Optimize and Improve the Teaching Environment

Optimizing and improving the teaching environment are an inevitable trend to strengthen and improve the effectiveness of ideological and political teaching in universities under the new situation. Therefore, ideological and political teachers should optimize and improve the teaching environment from multiple perspectives, eliminate negative factors as much as possible, and provide students with a harmonious, equal, and relaxed learning atmosphere. Marx has stressed that the environment is the main factor affecting human character, and it is reasonable to make the environment compatible with human nature. A harmonious environment has positive significance to the excavation and transformation of external factors of ideological and political teaching, plays a positive role in the development of the integration of direct and indirect teaching, and has an important influence on the enhancement of teaching integration, so civic and political science teachers should build learning contexts, cognitive contexts, and humanistic sensitization through multiple channels. Therefore, civic teachers should build learning contexts, cognitive contexts, and humanistic contexts through multiple channels to improve the effectiveness of ideological and political teaching while reflecting its charm.

## 6. Conclusions

In this study, the process of evaluating the teaching quality of college teachers as a system is studied from the perspective of input, output, information, and control of the system, and computer technology and mathematical methods are simultaneously applied as tools in the study of this problem of teaching quality in universities. Based on the survey questionnaire on the teaching quality of college teachers and the collection and analysis of survey data, the principle and method of the evaluation model of teaching quality of college teachers are elaborated based on the optimized BP neural network theory, and the software system of evaluation of teaching quality of college teachers is developed from the perspective of computer database development and program design. The software imported the survey data (including the comprehensive evaluation score of teaching quality and the evaluation score of its influencing factors) for the calculation of the teaching quality score, and compared and analyzed the calculated values of the test samples with the survey data values, and the degree of their conformity was quite good.

The results of the teacher teaching evaluation model based on an optimized neural network are very good, and the relative error is less than 10%, which indicated that it was practical to use the optimized BP neural network theory method for the analysis and calculation of teaching quality evaluation of college teachers.

## Figures and Tables

**Table 1:** Teaching quality evaluation index system of college teachers.

Primary indicators	Secondary indicators	Tertiary indicators
ITeacher teaching quality	I_1_ Instructional prerequisites	I_11_ Teachers' commitment and responsibility to teaching
		I_12_ Teachers' ability to teach and learn
		I_13_ Teachers' subject knowledge
		I_14_ Teachers' research achievements and research ability
	I_2_ Teaching process	I_21_ The scientific nature of teaching content and the effective information it contains
		I_22_ Reasonableness of teachers' teaching methods
		I_23_ The development of students' interest in learning
		I_24_ Whether the teacher has a suitable professional personality and teaching characteristics
		I_25_ Adaptability of teaching contents to students' needs
		I_26_ Teachers' compliance with school teaching regulations and discipline
	I_3_ Teaching effect	I_31_ The ideological, political, and moral qualities of students
		I_32_ Students' acquisition of basic professional knowledge and general knowledge
		I_33_ The improvement of students' practical and self-efficacy

**Table 2:** Results of teaching quality.

Number	Overall teaching quality score	Relative error (%)	Number	Overall teaching quality score	Relative error (%)
1	90	0	16	95.22	5.8
2	65.53	9.22	17	74.91	−0.12
3	77.17	2.89	18	47.4	5.33
4	81.36	8.48	19	81.91	9.21
5	98.26	9.18	20	64.17	6.95
6	64.84	8.07	21	60.79	1.32
7	81.55	8.73	22	65.08	8.47
8	60.57	0.95	23	81.12	8.16
9	80.14	6.85	24	92.67	2.97
10	74.44	−0.75	25	60.75	1.25
11	60.25	0.42	Inspection sample	63.96	6.6
12	48.66	8.13		77.94	3.96
13	60.62	1.03		82.15	9.53
14	60.85	1.42		60.85	1.42
15	60.95	1.58		61.22	2.03

## Data Availability

The data used to support the findings of this study are available from the corresponding author upon request.
